The article "Study on the Effect of Combination of Prednisone and Vitamin D in the Treatment of Primary Nephrotic Syndrome in Children" was retracted in 2023. Reason: concerns about the peer review.

# Study on the Effect of Combination of Prednisone and Vitamin D in the Treatment of Primary Nephrotic Syndrome in Children

**DOI:** 10.1155/2021/7932721

**Published:** 2021-10-12

**Authors:** Guoqun Zhou, Xiangdong Kong

**Affiliations:** ^1^Department of Pediatric, The First People's Hospital of Fuyang Hangzhou, Hangzhou 311400, Zhejiang, China; ^2^Department of Nephrology, The First People's Hospital of Fuyang Hangzhou, Hangzhou 311400, Zhejiang, China

## Abstract

**Objective:**

To study the effect of prednisone combined with vitamin D in the treatment of primary nephrotic syndrome in children.

**Method:**

73 cases of primary nephrotic syndrome admitted to the nephrology department of our hospital were randomly selected and retrospectively analyzed. 36 cases were treated with prednisone as the control group, and 37 cases were treated with prednisone combined with vitamin D as the observation group. The efficacy was compared after 3 months of continuous treatment.

**Result:**

After 3 months of treatment, the blood calcium of the observation group was higher than that of the control group, PTH was lower than that of the control group, and 25-(OH)2D3 and 1,25-(OH)2D3 were higher than those of the control group (*P* < 0.05). After 1, 2, and 3 months of treatment in the observation group, Scr and 24-h urine protein quantification were lower than those in the control group and eGFR was higher than that in the control group (*P* < 0.05). CD4+ and CD4+/CD8+ were lower in the observation group than in the control group after 3 months of treatment (*P* < 0.05). The serum sTfR and TGF-*β*1 levels were lower in the observation group than in the control group after 3 months of treatment (*P* < 0.05). The total effective rate of the observation group was 83.78% after 3 months of combined treatment with prednisone and vitamin D, which was significantly higher than the total effective rate of the control group of 61.11% (*P* < 0.05). The incidence of nausea and vomiting, heartburn, headache, dry cough, hypercalcemia, and constipation during treatment in the observation group was not statistically different from that in the control group (*P* > 0.05).

**Conclusion:**

Combined treatment of primary nephrotic syndrome in children with prednisone and vitamin D can more significantly improve the level of clinical indicators, improve renal function and immune function, and obtain more satisfactory efficacy, without significantly affecting the safety of treatment.

## 1. Introduction

Primary nephrotic syndrome is a group of nephropathies with a high incidence in the pediatric stage, mostly occurring in the glomerulus, and is a common manifestation of pediatric chronic kidney disease in which children are clinically hyperlipidemic and hypoalbuminemic, with massive proteinuria and varying degrees of edema [1]. Primary nephrotic syndrome is a group of autoimmune diseases, mostly mediated by immune damage. Abnormalities in humoral and cellular immune function and cytokine are closely linked to the development and progression of primary nephrotic syndrome [2].

Glucocorticoids have been the drug of choice for treating primary nephrotic syndrome and have been used in clinical treatment for a long time. The practice has shown that most pediatric primary nephrotic syndrome has a high sensitivity to glucocorticoid therapy and can achieve a satisfactory prognosis through treatment. However, some children still exhibit glucocorticoid resistance, which affects the efficacy and prognosis [3]. A study on risk factors for pediatric end-stage renal disease development showed that hormone-resistant nephrotic syndrome was an independent risk factor [4]. To ensure the clinical outcome, the combination of other drugs on top of glucocorticoids is proposed clinically, in addition to the choice of other highly sensitive glucocorticoids. Vitamin D is an essential drug for the clinical treatment of many diseases. Studies have found that vitamin D, especially active vitamin D3, has significant biological effects on cell proliferation, differentiation, and immune system regulation in various tissues [5].

However, there have been no previous studies on the treatment of primary nephrotic syndrome in children with prednisone combined with vitamin D. The efficacy and safety of combining these two drugs have not been confirmed. In this study, we specifically analyzed the difference in clinical effects between prednisone alone and combined with vitamin D in 73 children with primary nephrotic syndrome in order to explore more useful options for the pharmacological treatment of primary nephrotic syndrome in children.

## 2. Information and Method

### 2.1. Information

The case data of 73 children with primary nephrotic syndrome in the nephrology department of our hospital were retrospectively analyzed. In addition, all parents of the children were informed of the study and signed the study consent form. Also, the study was conducted through the ethical approval of the hospital where the study was conducted, and the ethical review approval number was 2021 LUN Research Approval No. 11.

Inclusion criteria: the age of children is under 12 years; children meet the diagnostic criteria of primary nephrotic syndrome [6]; children meet the indications for drug therapy; children are not receiving glucocorticoid therapy within the last 3 months; complete clinical case data; and children have stable condition.

Secondary nephrotic syndrome affects children. Also, secondary glomerulonephritis and inherited nephritis affect children. At the time of enrolment, children were still taking glucocorticoids. Antiepileptic medication usage in children is common. Drugs that are anticipated to be utilized in this research cause allergic responses in children. Children have concurrent participation in other studies. Children have comorbid psychiatric disorders or severe growth and development disorders.

## 3. Method

The children in both groups received the same basic symptomatic treatment and maintained a low-salt, low-fat, high-quality protein-rich diet. The control group was also treated with a single dose of prednisone, administered orally once a day, 1 mg/kg per dose, for 3 months. In the observation group, prednisone and vitamin D were combined and children were given prednisone tablets orally once a day at 1 mg/kg each time for 3 months and 300 IU of vitamin D (drug specification: 5000 units; approval number: State Drug Administration H33022361; manufacturer: Sanofi (Hangzhou) Pharmaceutical Co.).

### 3.1. Observed Indicators

General data: general data on age, sex, duration of disease, and type of pathology were collected for both groups.

Serum indexes: serum calcium, phosphorus, parathyroid hormone (PTH), 25-(OH)2D3, and 1,25-(OH)2D3 levels were measured before treatment and at the end of 3 months of treatment in both groups, respectively. Blood was collected from the upper limb two times in the morning under fasting condition and centrifuged at 4°C for 10 minutes at 3500 rpm. The assay kits were purchased from Shanghai Ruiqi Biotechnology Co, Ltd.

Renal function: 5 ml of venous blood was drawn from the child in fasting state, centrifuged for 5 minutes at 4°C and 3000 rpm, and the supernatant was stored at –20°C after centrifugation. The blood creatinine (Scr) level was measured by using an automatic biochemical analyzer, and the estimated glomerular filtration rate (eGFR) was calculated according to the MDRD formula: eGFR (ml/(min^*∗*^1.73 m^2^)) = 186 × (Scr)^−1.154^ × (age)^−0.203^ × 0.742 (if female), where Scr is serum creatinine, age is in years, and weight is in kg. In addition, the 24-hour urine following the child's first pee in the morning was kept, and the child's 24-hour urine protein quantity was evaluated using an automated biochemical analyzer. The test was performed four times: before therapy, one month after treatment, two months after treatment, and three months after treatment.

Immune function: 5 ml of venous blood was retained from both groups in the fasting state before and after 3 months of treatment, respectively, and processed by centrifugation at 4°C and 3000 rpm for 5 minutes continuously, and the levels of T lymphocyte subpopulations (CD4+, CD8+, and CD4+/CD8+) were measured by flow cytometry after retention of the supernatant. The kits procured by Roche were selected, and all operations were performed in strict accordance with the instructions.

Serum sTfR and TGF-*β*1 levels were measured: 5 ml of venous blood in the fasting state was taken as the test specimen before treatment and 3 months after treatment, respectively, and centrifuged at 4°C and 3000 rpm for 5 minutes continuously. The upper serum was retained, and then serum transferrin receptor (sTfR) and transforming growth factor-*β*1 (TGF-*β*1) levels were measured by using Beckman's fully automated enzyme immunoassay analyzer and the corresponding reagents from Roche.

Efficacy criteria [7]: complete remission: children with clinical symptoms disappeared after 3 months of treatment, renal function returned to normal, 24-h urine protein quantification less than 0.3 g, and blood creatinine and eGFR returned to normal or remained stable; partial remission: children with clinical symptoms disappeared after 3 months of treatment, renal function returned to normal, 24-h urine protein quantification between 0.3 and 1.0 g, and the blood creatinine and EGFR returned to normal or remained stable; no remission: children with no improvement in clinical symptoms after 3 months of treatment, kidney function still significantly abnormal or even continue to deteriorate, 24-h urine protein quantification more than 1.0 g, and blood creatinine and eGFR showed no change or were even worse than before. Total effective rate = complete remission rate + partial remission rate.

Treatment safety: compare the incidence of nausea and vomiting, heartburn, headache, dry cough, hypercalcemia, and constipation during treatment in both groups.

### 3.2. Statistical Method

All data were analyzed using SPSS 23.0, (*n* (%)) for count data by *X*^2^ test, ($\bar{x}$ ± *s*) for measurement data, *t*-test for independent samples for comparison between groups, paired *t*-test for intragroup pre-post comparisons, ANOVA analysis for multipoint comparisons, F-test, and GraphPad Prism 9 for graphs; *P* < 0.05 for statistical significance.

## 4. Result

### 4.1. General Information

The proportion of male versus female children, mean age, mean duration of disease, and each proportion of pathology type in the observation group showed no statistical difference compared with the control group (*P* > 0.05) (Table 1).

### 4.2. Serum Indicators

When compared between groups before treatment, the differences in serum calcium, phosphorus, PTH, 25-(OH)2D3, and 1,25-(OH)2D3 levels between the observation group and the control group were not statistically significant (*P* > 0.05); when compared between groups after 3 months of treatment, the differences in blood phosphorus between the two groups were not statistically significant (*P* > 0.05), the blood calcium in the observation group was higher than that in the control group, PTH was lower than that in the control group, and 25-(OH) 2D3 and 1,25-(OH)2D3 were higher than those in the control group (*P* < 0.05). Also, 1,25-(OH)2D3 were higher in the observation group than in the control group (*P* < 0.05); after 3 months of treatment, there was no significant difference in blood phosphorus between the observation group and the group before treatment (*P* > 0.05), blood calcium was higher than before treatment, PTH was lower than before treatment, and 25-(OH)2D3 and 1,25-(OH)2D3 were higher than before treatment (*P* < 0.05); after 3 months of treatment in the control group, blood phosphorus, blood calcium, and PTH were not statistically different from those before treatment (*P* > 0.05) and 25-(OH)2D3 and 1,25-(OH)2D3 were higher than before treatment (*P* > 0.05) (Figure 1).

### 4.3. Renal Function

When compared between groups before treatment, the differences in Scr, eGFR, and 24-h urine protein quantification between the observation group and the control group were not statistically significant (*P* > 0.05); when compared between groups after treatment, Scr and 24-h urine protein quantification in the observation group were lower than those in the control group after 1, 2, and 3 months of treatment and eGFR was higher than that in the control group (*P* < 0.05); Scr, eGFR, and 24-h urine protein quantification in the observation group were lower than those in the control group after 1, 2, and 3 months of therapy and eGFR was greater than before treatment (*P* < 0.05) when compared between groups before and after treatment. When comparing before and after treatment groups, Scr and 24-h urine protein quantification in the observation group were lower than before treatment and eGFR was higher than before treatment (*P* < 0.05). At the same time, there was no statistically significant difference between Scr, eGFR, and 24-h urine protein quantification in the control group after 1, 2, and 3 months of treatment and before treatment (*P* > 0.05) (Figure 2).

### 4.4. Immune Function

The differences in CD4+, CD8+, and CD4+/CD8+ levels between the two groups before treatment were not statistically significant (*P* > 0.05); after 3 months of treatment, CD4+ and CD4+/CD8+ in the observation group were lower than that in the control group (*P* < 0.05), and CD8+ was not significantly different from that in the control group (*P* > 0.05); when compared before and after treatment in the group, CD4+ and CD4+/CD8+ in the two groups after 3 months of treatment was lower than that in the control group (*P* < 0.05)and CD8+ was not significantly different from that in the control group (*P* > 0.05). CD8+ was lower than before treatment (*P* < 0.05), and the difference between CD8+ and before treatment was not significant (*P* > 0.05) (Figure 3).

### 4.5. Serum sTfR and TGF-*β*1 Level

The differences in serum sTfR and TGF-*β*1 levels between the two groups before treatment were not significant (*P* > 0.05); serum sTfR and TGF-*β*1 levels in the observation group were lower than those in the control group at the end of 3 months of treatment (*P* < 0.05); serum sTfR and TGF-*β*1 levels in both groups were lower after 3 months of treatment compared with those before treatment, and the differences were statistically significant (*P* > 0.05) (Figure 4).

### 4.6. Efficacy Criteria

After three months of combined prednisone and vitamin D therapy, the observation group's total effective rate was 83.78 percent, which was substantially greater than the control group's total effective rate of 61.11 percent (*P* < 0.05) (Table 2).

### 4.7. Treatment Safety

The incidence of nausea and vomiting, heartburn, headache, dry cough, hypercalcemia, and constipation during treatment in the observation group was not statistically different from that in the control group (*P* > 0.05) (Table 3).

## 5. Discussion

Pediatric nephrotic syndrome is a fibrotic lesion of the kidney caused by different factors, and most of them are primary. The blood of children with nephrotic syndrome is mostly in a hypercoagulable state, so the treatment needs to focus on anticoagulation. Glucocorticoids are widely used in the treatment of nephrotic syndrome. Prednisone is a typical glucocorticoid, and the application effect is widely confirmed. It, however, causes a variety of side effects, and clinical findings show that long-term use of the drug treatment will seriously stimulate the body's digestive tract, causing peptic ulcers, and even trigger hyperlipidemia, which will aggravate the hypercoagulable state of blood, causing more severe fibrosis in the tubular matrix of the child, leading to glomerulosclerosis. Therefore, it is important to actively explore other more effective and safe treatment options. Vitamin D is closely related to calcium and phosphorus metabolism and bone metabolism in the body, and 25-hydroxylase in the liver affects vitamin D3 to form 25-(OH)2D3, which is the highest level of circulating vitamin D metabolites in the body and can be used as an accurate indicator of vitamin D content in the body [8]. The blood circulating vitamin D metabolites bind to the hepatic vitamin D-specific transporter protein, which has the highest binding rate and affinity for 1,25-(OH)2D3 in particular [9]. In healthy individuals, vitamin D and metabolites bound to vitamin D-specific transporter proteins are not filtered by the glomerular filtration membrane, but in nephrotic syndrome because the glomerular filtration barrier is damaged, a large amount of protein-bound vitamin D and metabolites are lost in the urine, resulting in a significant decrease in circulating 25-(OH)2D3 levels and a corresponding decrease in 1,25-(OH)2D3 levels [10].

The difference in blood phosphorus between the two groups after 3 months of treatment in this study was not significant, but blood calcium, 25-(OH)2D3, and 1,25-(OH)2D3 were higher in the observation group than in the control group and PTH was lower than in the control group (*P* < 0.05), suggesting that combination drug therapy improved serum indicators more significantly and improved calcium and phosphorus metabolism as well as bone metabolism in the organism. It was found that children with primary nephrotic syndrome in remission who were sensitive to prednisone had significantly lower levels of 25-(OH)2D3 compared to healthy individuals, and no correlation was found between changes in this level and relapse status and disease duration [11]. Studies applying vitamin D in the treatment of primary nephrotic syndrome also showed a significant increase in 25-(OH)2D3 and 1,25-(OH)2D3 compared to the conventional treatment group [12]. Scr, 24-h urine protein quantification, and eGFR are useful indicators for clinical assessment of renal function. Studies have confirmed that, after the onset of nephrosis, Scr and 24-h urine protein quantification are abnormally elevated.

In contrast, eGFR will abnormally decrease, so controlling Scr and 24-h urine protein quantification levels and elevating eGFR levels can help improve renal function in children with nephrotic syndrome [13]. In this study, Scr and 24-h urine protein quantification were lower in the observation group than in the control group and eGFR was higher than in the control group after 1, 2, and 3 months of treatment (*P* < 0.05), which shows that combined treatment has a better effect on the improvement of renal function in children with primary nephrotic syndrome compared to glucocorticoid treatment alone. In addition, other studies have also shown that adjuvant application of vitamin D preparations in the treatment of pediatric primary nephrotic syndrome has an improvement in renal function [14].

As an autoimmune disease, immune function plays an essential role in developing and progressing primary nephrotic syndrome [15]. It was found that the majority of children with nephropathy have significantly disturbed immune function, which was analyzed as a result of T-lymphocyte subsets that affect the immune status of the organism. It is believed that the immune function of children with nephropathy can be assessed. The efficacy of the treatment can be determined by measuring the level of T-lymphocyte subsets [16]. In this study, CD8+ did not differ significantly from the control group after 3 months of treatment, but CD4+ and CD4+/CD8+ were lower than in the control group, suggesting that combined treatment with vitamin D regulates the body's immune function more substantially than single application of prednisone treatment. CD4+ and CD8+ are the two main subpopulations of T lymphocytes, and CD4+ is a participant in B lymphocyte differentiation and antibody production, as well as CD4+ is a participant in the cell-mediated immune response, while CD8+ is a suppressor of T lymphocytes and helps in the elimination of pathogens [17, 18]. CD4+/CD8+ reflects the immune status of the body and regulates the body's immune response, playing an important role in maintaining the stability of the immune state [19]. After 3 months of therapy, serum sTfR and TGF-*β*1 levels in the observation group were lower than those in the control group (*P* > 0.05). Increased levels of sTfR may increase inflammatory responses or fibrotic changes in the disease [20]. It belongs to a group of transmembrane proteins that have a major effect on the development, progression, and reversal of kidney disease. TGF-*β*1 is a peptide that regulates cell growth and cell differentiation and is important for stable kidney function and structural stability. It is important for the maintenance of functional stability and structural stability of the kidney [21]. In primary nephrotic syndrome, TGF-*β*1 accelerates the synthesis of extracellular matrix such as fibroblasts and inhibits the degradation of extracellular matrix components, thus accelerating glomerulosclerosis and interstitial fibrosis [22, 23], so it is important to control its level to reduce the condition of nephrosis and improve the renal function of children with nephrosis.

In conclusion, the combination of prednisone and vitamin D for the treatment of primary nephrotic syndrome in children can more significantly improve the level of clinical indicators, improve renal function and immune function, and obtain more satisfactory efficacy, without significantly affecting the safety of treatment.

## Figures and Tables

**Figure 1:** Compared with the control group before treatment, the differences in serum calcium (a), phosphorus (b), PTH (c), 25-(OH)2D3 (d), and 1,25-(OH)2D3 (e) levels in the observation group were not statistically significant (*P* > 0.05); compared with the control group after 3 months of treatment, PTH in the observation group was lower than that in the control group, blood calcium, 25-(OH)2D3, and 1,25-(OH)2D3 were higher than those in the control group (*P* < 0.05), and the difference in blood phosphorus was not statistically significant (*P* > 0.05); compared with the groups before treatment, after 3 months of therapy, there was no significant change in blood phosphorus in the observation group (*P* > 0.05), PTH was lower than before treatment and blood calcium, 25-(OH)2D3, and 1,25-(OH)2D3 were higher than those before treatment (*P* < 0.05). However, the results for the control group were as follows: there was no statistical difference in blood phosphorus, blood calcium, and PTH after 3 months of treatment (*P* > 0.05), and 25-(OH)2D3 and 1,25-(OH)2D3 were higher than before treatment (*P* > 0.05).

**Figure 2:** Compared with the levels of Scr (a), 24-h UTP (b), and eGFR (c) before treatment in the control group, there was no significant difference in the observation group (*P* > 0.05). Compared with the control group after 1, 2, and 3 months of treatment, the levels of Scr (a) and 24-h UTP (b) were lower and the levels of eGFR (c) were higher in the observation group (*P* < 0.05).

**Figure 3:** Compared with the control group before treatment, CD4+ (a), CD8+ (b), and CD4+/CD8+ (c) levels, there was no significant difference in the observation group (*P* > 0.05); compared with the control group after 3 months of treatment, the observation group CD4+ and CD4+/CD8+ levels were lower (*P* < 0.05) and CD8+ difference was not significant (*P* > 0.05). Compared with the group before treatment, CD4+ (a) and CD4+/CD8+ (c) were lower after 3 months of treatment (*P* < 0.05) and the difference in CD8+ (b) was insignificant (*P* > 0.05).

**Figure 4:** Compared with the sTfR (a) and TGF-*β*1 (b) levels before treatment in the control group, there was no significant difference in the observation group (*P* > 0.05), and compared with the sTfR and TGF-*β*1 levels after 3 months of treatment in the control group, both were lower in the observation group (*P* < 0.05).

**Table 1:** Comparison of general information between the 2 groups ($\bar{x}$ ± *s*)/(*n* (%)).

Information		Observation group (*n* = 37)	Control group (*n* = 36)	t/X^2^	*P*
Gender	Male	20 (54.05)	21 (58.33)	0.136	0.713
	Female	17 (45.95)	15 (41.67)		

Age (years)		7.12 ± 3.92	7.55 ± 4.12	0.457	0.649

Duration of illness (months)		7.75 ± 1.04	7.79 ± 1.06	0.163	0.871

Type of pathology	Focal segmental glomerulosclerosis	10 (27.03)	9 (25.00)	0.519	0.327
	Thylakoid proliferative glomerulonephritis	11 (29.73)	12 (33.33)		
	Membranoproliferative glomerulonephritis	14 (37.84)	12 (33.33)		
	Others	2 (5.41)	3 (8.33)		

**Table 2:** Comparison of the total effective rate after 3 months of treatment between the two groups (*n* (%)).

Grouping	Complete relief	Partial relief	No relief	Total efficiency
Observation group (*n* = 37)	13 (35.14)	18 (48.65)	6 (16.22)	31 (83.78)
Control group (*n* = 36)	10 (27.78)	12 (33.33)	14 (38.89)	22 (61.11)
*X* ^2^				4.716
*P*				0.030

**Table 3:** Comparison of the incidence of adverse reactions during treatment between the two groups (*n* (%)).

Grouping	Nausea and vomiting	Heartburn	Headaches	Dry cough	Hypercalcemia	Constipation
Observation group (*n* = 37)	4 (10.81)	2 (5.41)	1 (2.70)	2 (5.41)	1 (2.70)	2 (5.41)
Control group (*n* = 36)	3 (8.33)	3 (8.33)	1 (2.78)	2 (5.56)	2 (5.56)	3 (8.33)
*X* ^2^	0.002	0.001	0.486	0.236	0.001	0.001
*P*	0.970	0.975	0.486	0.627	0.981	0.975

## Data Availability

The data used to support the findings of this study are included within the article.
